The article "Ovarian Cancer Risk Scores Based on Immune-Related Pseudogenes to Predict Overall Survival and Guide Immunotherapy and Chemotherapy" was retracted in 2023. Reasons: unreliable results or conclusions; concerns about the data; concerns about the peer review; concerns about the citations.

# Ovarian Cancer Risk Scores Based on Immune-Related Pseudogenes to Predict Overall Survival and Guide Immunotherapy and Chemotherapy

**DOI:** 10.1155/2021/1586312

**Published:** 2021-10-08

**Authors:** Jie Zhao, Rixiang Zhao, Xiaocen Wei, Xiaojing Jiang, Fan Su

**Affiliations:** Oncology Department, Laixi People's Hospital of Shandong Province, Qingdao, China

## Abstract

**Background:**

Ovarian cancer (OC) is the top of the aggressive malignancies in females with a poor survival rate. However, the roles of immune-related pseudogenes (irPseus) in the immune infiltration of OC and the impact on overall survival (OS) have not been adequately studied. Therefore, this study aims to identify a novel model constructed by irPseus to predict OS in OC and to determine its significance in immunotherapy and chemotherapy.

**Methods:**

In this study, with the use of The Cancer Genome Atlas (TCGA) combined with Genotype-Tissue Expression (GTEx), 55 differentially expressed irPseus (DEirPseus) were identified. Then, we constructed 10 irPseus pairs with the help of univariate, Lasso, and multivariate Cox regression analysis. The prognostic performance of the model was determined and measured by the Kaplan–Meier curve, a time-dependent receiver operating characteristic (ROC) curve.

**Results:**

After dividing OC subjects into high- and low-risk subgroups via the cut-off point, it was revealed that subjects in the high-risk group had a shorter OS. The multivariate Cox regression performed between the model and multiple clinicopathological variables revealed that the model could effectively and independently predict the prognosis of OC. The prognostic model characterized infiltration by various kinds of immune cells and demonstrated the immunotherapy response of subjects with cytotoxic lymphocyte antigen 4 (CTLA4), anti-programmed death-1 (PD-1), and anti-PD-ligand 1 (PD-L1) therapy. A high risk score was related to a higher inhibitory concentration (IC_50_) for etoposide (*P*=0.0099) and mitomycin C (*P*=0.0013).

**Conclusion:**

It was the first study to identify a novel signature developed by DEirPseus pairs and verify the role in predicting OS, immune infiltrates, immunotherapy, and chemosensitivity. The irPseus are vital factors predicting the prognosis of OC and could act as a novel potential treatment target.

## 1. Introduction

Ovarian cancer (OC) is a common highly aggressive malignancy of the female reproductive system, with the 4th highest morbidity and the 3rd highest mortality around the world [1]. The report of Global Cancer Statistics 2020 estimated that the incidence and mortality of OC accounts for 1.6% and 2.1%, respectively [2]. The current regular treatment strategy for OC is to quickly resect the primary lesion or followed by adjuvant chemotherapy. Recently, an open-label, randomized, phase 3 trial investigated progression-free survival and incidence of adverse events after chemotherapy with or without avelumab followed by avelumab maintenance versus chemotherapy alone in 998 patients with previously untreated epithelial OC, while the results failed to support the use of avelumab in the frontline treatment setting [3]. Increasing evidence demonstrated that tumor microenvironments and immune cell infiltration play vital roles during the process of malignancies development and treatment [4]. The increasing reports demonstrated that immunotherapy is developing as a promising treatment strategy in malignancy therapy. Multiple studies demonstrated the performance of immunotherapy, such as spontaneous cancer regressions in OC and revealed the possible procedures of immune evasion and responses to immune checkpoint inhibitors in patients with OC [5–7]. However, a recent placebo-controlled randomized phase III trial failed to support the clinical use of immune checkpoint inhibitors such as atezolizumab and bevacizumab in newly diagnosed OC [8]. Pseudogenes, belonging to a subgroup of long noncoding RNAs, were firstly labeled as nonfunctional “gene fossils” or “junk genes,” but recent studies have showed their involvement in many biological functions, including tumor progression and prognosis [9–11]. Accumulating evidence revealed that pseudogenes manifest functional roles. As we have known, pseudogene-related lncRNAs have been demonstrated to adjust their parent genes and the new discovered mechanism has been noted in various cancer kinds, including OC [12, 13]. Some tumor-related pseudogenes can be utilized as predictors of prognosis. It was reported that high expression of RP11-564D11.3 was associated with adverse prognosis in hepatocellular carcinoma [14]. Pseudogenes can control gene expression at transcriptional and post-transcriptional levels. It was reported that MYC can result in oncogenesis via transcriptional supervision of HMGA1P6 in OC [13]. However, the generally predictive significances of irPseus in OC have not been fully studied and the probable significances of pseudogenes in OC remain uncertain. Therefore, for the first time, we developed an irPseus signature in OC to predict OS and guide immunotherapy and chemotherapy.

We adopted a new pairwise algorithm to develop an irPseus pair signature without requiring the exact expression values [15, 16]. Next, we explored its predictive significance among individuals with OC, as well as chemotherapeutic efficacy, and tumor immune infiltration. We firstly identified 55 differentially expressed irPseus (DEirPseus) via transcriptomic matrix analysis in OC compared with normal tissues from GTEx, and 424 irPseus pairs were created. Then, by univariate regression, we screened OS-related irPseus pairs. Next, we narrowed down the pairs by LASSO algorithm and multivariate regression, from which we developed a 10-irPseus pair-based prognostic model.

## 2. Methods

### 2.1. Data Collection and Immune Genes and Pseudogenes Sources

We downloaded and further analyzed the mRNA expression matrix of 379 OC samples from TCGA cohorts via UCSC Xena (http://xena.ucsc.edu/) and from 88 normal ovarian tissues by the GTEx portal (https://www.gtexportal.org). The corresponding clinical data were used for survival investigation. The two portals are publicly available databases without requiring ethical review approval. A total of 1793 immune-related genes were collected and downloaded via the ImmPort portal (https://immport.niaid.nih.gov). Next, 13602 pseudogenes were picked up through the HGNC database (https://www.genenames.org/). The Spearman correlation analysis was then utilized to label the irPseus between the immune genes and pseudogenes if they met the following criteria: |correlation coefficient| > 0.6 and *P* < 0.001.

### 2.2. Identification of DEirPseus and irPseus Pairs Establishment

The “limma” package in *R* along with normalization strategies was used to combine the gene expression matrixes from TCGA and GTEx portals and compute DEirPseus between OC and normal tissues. A false discovery rate (FDR) ≤ 0.05 and |log2(fold change)| ≥ 1 were used as the threshold value. Next, we developed possible pseudogene pairs based on the DEirPseus. In a gene pair, two genes established a pseudogene pair in alphabetical order. If the expression value of the former is larger than the latter, the pseudogene pair yielded a score of 1; otherwise, the score was 0.

### 2.3. Prognostic Signature Construction

All pseudogene pairs developed were used as the candidate variables for prognosis signature construction. Next, we adopted the univariate Cox regression model to identify prognosis-associated pseudogene pairs that were notably associated with OS (*P* < 0.05). To prevent overfitting in the model, we further simplify the model. Next, the range of gene pairs was further reduced while maintaining high accuracy using the LASSO regression analysis with 10-fold cross-validation. It selects variables and evaluates parameters altogether and better solves the multicollinearity puzzle and controls the complexity of the model in regression analysis [17]. Finally, a Cox proportional hazards model together with the stepwise algorithm was performed to develop a prognostic signature. Every patient received an individual risk score using the following formula: Risk score = Expression of irPseus pair_1_ *∗* *β*irPseus pair_1_ + Expression of irPseus pair_2_ *∗* *β*irPseus pair_2_ + ⋯ + Expression of irPseus pair_*n*_ *∗* *β*irPseus pair_*n*_, in which *n* is the number of pseudogene pairs and *β* indicates the regression coefficient obtained through the multivariate Cox regression algorithm. Based on the individual risk scores, all subjects were separated into high- and low-risk subgroups, according to the best cut-off of the risk scores established by time-dependent ROC curves at 1-year OS.

### 2.4. Validating the Performance of the Prognostic Model

The survival differences between the two groups were explored via the Kaplan–Meier survival curve along with the log-rank test. In addition, the accuracy of prognostic model was detected by ROC curve analysis and computed by the AUC in 1, 3, and 5 years. In addition, multivariate Cox regression analyses were conducted to confirm whether the risk score can independently predict the OS of patients with OC among other clinicopathological features.

### 2.5. Tumor-Infiltrating Immune Cells and Their Association with the Model

To examine the link between the risk score and tumor-infiltrating immune cells, we included several algorithms to compute the immune infiltration levels in the OC patients, including CIBERSORT, XCELL, TIMER, EPIC, MCPcounter, and QUANTISEQ. The discrepancy in immune infiltrating cell proportion calculated by the above algorithms between high- and low-risk subgroups of the developed signature was examined by the Wilcoxon signed-rank test. The possible link between the signature risk score and the immune infiltrated cells was conducted using the Spearman correlation analysis and was visualized via a lollipop diagram.

### 2.6. Analyses of the Signature Risk Score and the Immune Checkpoint Inhibitor Genes

Immune checkpoint inhibition has become an effective and wide-used method of immunotherapy. Substantial breakthrough advances have been acquired in the understanding of immune surveillance, including the possible mechanism of PD-1, PD-L1, and CTLA4 in the progression of cancers. To explore the link between the signature risk score and the expression level of immune checkpoint inhibitor genes, we used the ggstatsplot package and violin plot to display the relationship.

### 2.7. Examination of the Value of the Signature in the Chemotherapeutics

To investigate the signature for the therapy of OC, the IC_50_ of generally using chemotherapeutic medication, such as etoposide, mitomycin, and cisplatin, in the OC cohort was computed via the Wilcoxon signed-rank test.

### 2.8. Statistical Analysis

The difference of various clinicopathological variables was compared between two groups by Student's *t*-tests. The multivariate Cox regression was carried out via *R* package “survival” along with hazard ratios (HRs) and 95% confidence intervals (CIs). A *P* < 0.05 indicated statistical significance. Time-dependent ROC curves were plotted using the “pROC” package. All the statistical analyses in this study were performed using *R* software, version 3.6.1 (https://www.r-project.org/).

## 3. Results

### 3.1. Identification of Pairwise Pseudogenes and Construction of the Prognostic irPseus Pair Model

A total of 97 irPseus were identified via the Spearman correlation analysis. We identified 55 DEirPseus (Figure 1(a)), among which 39 pseudogenes were upregulated and 16 pseudogenes were downregulated (Figure 1(b)). A total of 369 OC individuals were matched with their corresponding complete survival information. Based on the pseudogenes pair algorithm, 424 irPseus pairs were created. Univariate Cox regression analysis was firstly utilized for the screening of OS-related pseudogenes, and 54 prognostic irPseus pairs were identified. Next, we carried out the LASSO algorithm after 1000 iterations to shrink the count of variables in the risk signature (Figure 2(a) and 2(b)), and totally 10 irPseus pairs were identified (Figure 2(c)) using multivariate Cox regression analysis, which included 18 pseudogenes. The risk score was developed based on the expression patterns of these pairwise irPseus weighted by their correspondence coefficient received from multivariate Cox regression. Therefore, the risk score was computed for all patients. Then, we computed the AUCs for each ROC curve of 10 irPseus pairs, plotted the curved line, and demonstrated the optimal point locating at 1.204 to identify the most optimal irPseus pair for the maximum AUC value (Figure 3(a)). To further confirm the optimality, we firstly draw a 1-year ROC curve, which indicated the AUC value was larger than 0.75 (Figure 3(b)). As for 2- and 3-year AUCs, the values were 0.744 and 0.697, respectively (Figure 3(c)). Furthermore, we analyzed the 1-year ROC curves with previous clinical pathological variables such as age, grade, clinical stage, and neoplasm. It was revealed that the AUC value of the irPseus pairs signature was 0.759, which was higher than the AUC values for age (AUC = 0.712), grade (AUC = 0.541), clinical stage (AUC = 0.591), and neoplasm (AUC = 0.585), as shown in Figure 3(d).

### 3.2. The irPseus Pair Model Risk Score as Independent Prognostic Factors for OC

The optimal cut-off of the risk score determined in the TCGA cohort was used to re-distinguish individuals into the high- and low-risk subgroups. The model risk score distribution and patients' survival condition of each individual are displayed in Figure 4(a) and 4(b). The novel irPseus pair model could divide OC individuals into low- and high-risk subgroups with distinct OS and elevated risk score indicating a higher possibility of mortality (Figure 4(c)).

Then, we conducted several chi-square and Wilcoxon signed-rank tests to explore the possible link between the risk of OC and clinicopathological variables. It was revealed that age (Figure 5(a)), survival status (Figure 5(b)), and neoplasm status (Figure 5(c)) were strikingly associated with the signature risk score, while stage (Figure 5(d)) and grade (Figure 5(e)) were not associated with the signature risk score (all *P* > 0.05).

Furthermore, we adapted univariate and multivariable Cox regression analyses to test if the irPseus pair model risk score could serve as an independent prognostic variable. We confirmed that age (HR = 1.017, 95% CI = 1.002–1.033, *P* = 0.025), neoplasm status (HR = 6.257, 95% CI = 3.185–12.294, *P* < 0.001), and risk score (HR = 2.193, 95% CI = 1.745–2.756, *P* < 0.001) exhibited obvious statistical differences with the help of univariate Cox regression analysis (Figures 5(f) and 5(g)). The multivariate Cox regression analysis revealed risk score (HR = 1.932, 95% CI = 1.530–2.439, *P* < 0.001) and neoplasm status (HR = 5.477, 95% CI = 2.771–10.825, *P* < 0.001) as independent prognostic factors for OC.

### 3.3. Association between the irPseus Pair Signature, Tumor-Infiltrating Immune Cells, and Immune Checkpoint Inhibitors

To explore the differences of immune cell abundance between high- and low-risk subgroups, we consequently measured the relationship between the signature and the tumor immune microenvironment via the Wilcoxon signed-rank test. We concluded that the signature risk score was mainly involved in tumor-infiltrating immune cells such as B cell, macrophage, macrophage M1, plasmacytoid dendritic cell, macrophage M2, cancer-associated fibroblast, CD8^+^ T cell, endothelial cell, neutrophil, stroma score, uncharacterized cell, NK cell, CD4^+^ T cell, and T cell follicular helper (Figure S1). A detailed Spearman correlation analysis was carried out and is presented in Figure 6(a). The appearance of immune checkpoint inhibitors in recent years has revolutionized the therapeutic mode of cancer individuals. Immune checkpoint inhibition has become an effective and wide-used method of immunotherapy. We examined if the signature risk score was associated with immune checkpoint inhibitor genes and demonstrated that the model high risk scores were negatively associated with high expression of CTLA4 (*P* < 0.01, Figure 6(b)), PD-1 (*P* < 0.001, Figure 6(c)), and PD-L1 (*P* < 0.001, Figure 6(d)).

### 3.4. Association between the irPseus Pair Signature and Chemotherapeutics

In addition to checkpoint blockades treatment, we also aimed to study associations between irPseus pair signature and the performance of conventional chemotherapeutics in treating OC. It was revealed that a high risk score was closely related to a higher half IC_50_ of chemotherapeutics, such as etoposide (*P*=0.0099) and mitomycin (*P*=0.0013), whereas the relationship failed to be statistically significant for cisplatin (*P*=0.072, Figure 6(e)–6(g)), which demonstrated that the irPseus pairs signature served as a potential factor for chemosensitivity in OC.

## 4. Discussion

OC is still a common gynecological malignancy with a heterogeneous category that seriously threatens a woman's health. As a progressive disease, OC requires robust biomarkers and models to forecast the outcome and therapeutic targets. With the rapid progression of gene sequencing technology, mRNA expression-based prognostic signatures are being served as an approach to evaluate tumor progression. Nevertheless, majority of these models relayed on mRNAs or gene-quantifying expression [18–20]. In our study, for the first time, we used the strategy of irPseus pairs pairing and aimed to develop a reliable signature with 10-pseudogene combinations and not requiring specific expression levels of the pseudogene.

First, we extracted the pseudogenes expression matrix from TCGA and conducted a differential coexpression analysis using the Spearman correlation analysis to identify DEirPseus and created irPseus pairs using a novel method of relative expression orders matrix. Second, we carried out univariate analysis, LASSO, and multivariate Cox regression to identify prognostic-related irPseus pairs. Finally, we assessed the novel irPseus signature under several clinical backgrounds, including OS, clinical factors, tumor-infiltrating immune cells, checkpoint-related molecules, and chemosensitivity.

Increasing evidence indicated that the immune system plays a vital role in malignancy initiation, cancer progression, and cancer therapeutic responses. Immune cells have been confirmed to have a significant influence on various disease processes, including cancer progression [21–23]. So far, immunotherapies in OC are remaining in the exploratory stages. Nevertheless, a growing number of *in vitro* and *in vivo* clinical immunotherapies have been performed. We further analyzed the infiltration level of immune cells between two risk subgroups. It has been confirmed that macrophages are vital immune cells that closely took part in inflammation and tumorigenesis [24]. Macrophages that infiltrate around various tumor cells are named tumor-associated macrophages, which included antitumor M1 macrophages and tumor-promoting M2 macrophages [25]. Moreover, a previous study has confirmed that a large M1/M2 ratio of TAM was closely related to prolong OS in OC patients [26]. M2 macrophages could produce immunosuppressive events to contribute to immune escape of OC [27]. In our study, CD8+ T cell, T cell follicular helper, and CD4+ T cell also showed obvious differences between two risk groups. OC was known as one of the immunogenic cancers that responded pretty well via targeting the immune checkpoints [28]. It has verified that joined CTLA4 antibody and poly ADP-ribose polymerase inhibitor therapy in BRCA1-deficient OC individuals greatly extended OS mediated by T cells [29]. Neutrophils were notably related to poor survival among the high-grade OC individuals (HR: 1.14–1.73) [30]. A recent report revealed that eosinophils, neutrophils, and T cell follicular helper were obviously involved in OC survival [31]. A 17 transcription factors-based prognostic signature revealed that B cells, NK cells, and T cells were confirmed to be different between the two groups, and individuals in the low-risk subgroup were more cline to response to immunotherapy and chemotherapy including etoposide, paclitaxel, and veliparib. In this study, we revealed that a low risk score was closely related to a higher half IC_50_ of etoposide and mitomycin. Based on the above findings, the irPseus involved in the model play a vital role in human OC.

The novel algorithm used in this study had several strengths. First, traditional approaches previous studies used only focused on each gene independently using gene expression levels among different data sets that requiring scaling and appropriate normalization, which posed a highly formidable challenge owing to the potential biological heterogeneity between different platforms. We adapted a new algorithm for the identification of functional links between pairwise irPseus via relative expression orderings of two irPseus within-sample absence of the need of the above requirements. Second, the cut-off of the risk score can be directly used to other external validation groups since it was calculated based on expression values (0 or 1) of the pairwise irPseus weighted by their relative coefficient. Third, our study focused on identifying prognostic pairwise irPseus rather than multiple prognostic pseudogenes, and this algorithm can identify prognostic irPseus pairs from mRNA expression profiles although some pseudogenes do not show significant prognostic value. However, the study has limitations. First, our research is based on large-scale OC data sets in a public database and the conclusions were not confirmed by an external independent cohort. Second, the functions of the pseudogenes that make up the irPseus pairs have not been verified, and future biological experiments are required to elaborate the possible functional mechanism in OC.

In summary, we established a new 10-irPseus pair model for OC, which is a promising prognostic factor and can act as a vital biomarker for predicting the OS of patients with OC and helping in distinguishing individuals who may benefit from chemotherapeutics and immunotherapy.

## Figures and Tables

**Figure 1:** Differentially expressed immune-related pseudogenes in ovarian cancer. (a) Expression levels of 55 immune-related pseudogenes in OC tissues and normal tissues are presented in the heatmap; blue color to red color indicates downregulation to upregulation. (b) All immune-related pseudogenes explored in OC are displayed via the volcano plot.

**Figure 2:** Immune-related pseudogenes pairs identification and signature construction. (a) LASSO regression of the 55 OS-related immune-related pseudogenes pairs. (b) 10-fold cross-validation for adjusting the pseudogenes pair selection using the LASSO regression. (c) Signature construction via multivariable Cox regression analyses.

**Figure 3:** Evaluation of a new prognostic model by immune-related pseudogenes pairs. (a) Seeking the highest point of the AUC via the optimal cut-off of the signature. (b) The ROC of the best irPseus pair signature was associated with the maximum AUC value. (c) The 1-, 3-, and 5-year ROC curves of the irPseus pair signature. (d) A detailed comparison of 1-year AUC values with more generally used variables demonstrated the superiority of the irPseus pair signature risk score.

**Figure 4:** Performance of the irPseus pair signature for prognosis prediction. (a) The 10-irPseus pair model and its risk score distribution status and (b) patients survival outcome status. (c) Individuals in the high-risk subgroup presented a shorter OS revealed by the Kaplan–Meier test.

**Figure 5:** Clinical performance of the irPseus pair signature. The scatter diagram demonstrated the relationships between signature risk score and multiple clinicopathological factors (a) age, (b) survival status, (c) neoplasm status, (d) clinical stage, and (e) tumor grade. (f) Univariate and (g) multivariate analyses were carried out to seek the independent prognostic characteristics.

**Figure 6:** Evaluation of tumor-infiltrating immune cells and immune checkpoint inhibitor genes with signature. (a) Patients in the two risk groups showed a close link between tumor-infiltrating immune cells and the model revealed by Spearman correlation analysis. Low risk scores of the model were positively related to upregulated (b) CTLA4, (c) PD-1, and (d) PD-L1 expressions in patients with OC. (e), (f), and (g) The irPseus pair signature served as a possible tool for chemosensitivity since low risk scores were obviously involved in a higher IC_50_ for chemotherapeutics, such as etoposide and mitomycin. ^*∗∗∗*^*P* < 0.001.

## Data Availability

The data used in the study can be downloaded from TCGA (https://www.cancer.gov/about-nci/organization/ccg/research/structural-genomics/tcga), the ImmPort (https://immport.niaid.nih.gov), and the HGNC database (https://www.genenames.org/).

## Supplementary Materials

Supplementary Materials Figure S1. The main results of the assessment of tumor-infiltrating immune cells with irPseus pair signature.

## References

[1] Bray F., Ferlay J., Soerjomataram I., Siegel R. L., Torre L. A., Jemal A. (2018). Global cancer statistics 2018: GLOBOCAN estimates of incidence and mortality worldwide for 36 cancers in 185 countries. *CA: A Cancer Journal for Clinicians*.

[2] Sung H., Ferlay J., Siegel R. L. (2021). Global cancer statistics 2020: GLOBOCAN estimates of incidence and mortality worldwide for 36 cancers in 185 countries. *CA: A Cancer Journal for Clinicians*.

[3] Monk B. J., Colombo N., Oza A. M. (2021). Chemotherapy with or without avelumab followed by avelumab maintenance versus chemotherapy alone in patients with previously untreated epithelial ovarian cancer (JAVELIN Ovarian 100): an open-label, randomised, phase 3 trial. *The Lancet Oncology*.

[4] Anandappa A. J., Wu C. J., Ott P. A. (2020). Directing traffic: how to effectively drive T cells into tumors. *Cancer Discovery*.

[5] Schlienger K., Chu C. S., Woo E. Y. (2003). TRANCE- and CD40 ligand-matured dendritic cells reveal MHC class I-restricted T cells specific for autologous tumor in late-stage ovarian cancer patients. *Clinical Cancer Research: An Official Journal of the American Association for Cancer Research*.

[6] Goodell V., Salazar L. G., Urban N. (2006). Antibody immunity to the p53 oncogenic protein is a prognostic indicator in ovarian cancer. *Journal of Clinical Oncology*.

[7] Oda K., Hamanishi J., Matsuo K., Hasegawa K. (2018). Genomics to immunotherapy of ovarian clear cell carcinoma: unique opportunities for management. *Gynecologic Oncology*.

[8] Moore K. N., Bookman M., Sehouli J. (2021). Atezolizumab, bevacizumab, and chemotherapy for newly diagnosed stage III or IV ovarian cancer: placebo-controlled randomized phase III trial (IMagyn050/GOG 3015/ENGOT-OV39). *Journal of Clinical Oncology*.

[9] The ENCODE Project Consortium (2012). An integrated encyclopedia of DNA elements in the human genome. *Nature*.

[10] Tang S., Zhuge Y. (2021). An immune-related pseudogene signature to improve prognosis prediction of endometrial carcinoma patients. *BioMedical Engineering Online*.

[11] Du Y., Gao Y. (2020). Development and validation of a novel pseudogene pair-based prognostic signature for prediction of overall survival in patients with hepatocellular carcinoma. *BMC Cancer*.

[12] Kubiczak M., Walkowiak G., Nowak-Markwitz E., Jankowska A. (2013). Human chorionic gonadotropin beta subunit genes CGB1 and CGB2 are transcriptionally active in ovarian cancer. *International Journal of Molecular Sciences*.

[13] Tian X., Song J., Zhang X. (2020). MYC-regulated pseudogene HMGA1P6 promotes ovarian cancer malignancy via augmenting the oncogenic HMGA1/2. *Cell Death & Disease*.

[14] Song H., Yang J., Zhang Y., Zhou J., Li Y., Hao X. (2019). Integrated analysis of pseudogene RP11-564D11.3 expression and its potential roles in hepatocellular carcinoma. *Epigenomics*.

[15] Heinäniemi M., Nykter M., Kramer R. (2013). Gene-pair expression signatures reveal lineage control. *Nature Methods*.

[16] Zhao E., Chen S., Dang Y. (2021). A novel signature based on pairwise PD-1/PD-L1 signaling pathway genes for predicting the overall survival in patients with hepatocellular carcinoma. *Clinical and Translational Medicine*.

[17] Duan J., Soussen C., Brie D., Idier J., Wan M., Wang Y.-P. (2016). Generalized LASSO with under-determined regularization matrices. *Signal Processing*.

[18] Yu Z., He H., Chen Y., Ji Q., Sun M. (2021). A novel ferroptosis related gene signature is associated with prognosis in patients with ovarian serous cystadenocarcinoma. *Scientific Reports*.

[19] Zhang Y., Liu J., Raj-Kumar P.-K. (2020). Development and validation of prognostic gene signature for basal-like breast cancer and high-grade serous ovarian cancer. *Breast Cancer Research and Treatment*.

[20] Ye Y., Dai Q., Qi H. (2021). A novel defined pyroptosis-related gene signature for predicting the prognosis of ovarian cancer. *Cell Death Discovery*.

[21] Liu J., Meng H., Nie S. (2020). Identification of a prognostic signature of epithelial ovarian cancer based on tumor immune microenvironment exploration. *Genomics*.

[22] Zhao E., Xie H., Zhang Y. (2020). Predicting diagnostic gene biomarkers associated with immune infiltration in patients with acute myocardial infarction. *Frontiers in Cardiovascular Medicine*.

[23] Zuo S., Wei M., Wang S., Dong J., Wei J. (2020). Pan-cancer analysis of immune cell infiltration identifies a prognostic immune-cell characteristic score (ICCS) in lung adenocarcinoma. *Frontiers in Immunology*.

[24] Grivennikov S. I., Greten F. R., Karin M. (2010). Immunity, inflammation, and cancer. *Cell*.

[25] Sica A. (2010). Role of tumour-associated macrophages in cancer-related inflammation. *Experimental Oncology*.

[26] Zhang M., He Y., Sun X. (2014). A high M1/M2 ratio of tumor-associated macrophages is associated with extended survival in ovarian cancer patients. *Journal of Ovarian Research*.

[27] Cheng H., Wang Z., Fu L., Xu T. (2019). Macrophage polarization in the development and progression of ovarian cancers: an overview. *Frontiers in Oncology*.

[28] Ghisoni E., Imbimbo M., Zimmermann S., Valabrega G. (2019). Ovarian cancer immunotherapy: turning up the heat. *International Journal of Molecular Sciences*.

[29] Higuchi T., Flies D. B., Marjon N. A. (2015). CTLA-4 blockade synergizes therapeutically with PARP inhibition in BRCA1-deficient ovarian cancer. *Cancer Immunology Research*.

[30] Gao Y., Chen L., Cai G. (2020). Heterogeneity of immune microenvironment in ovarian cancer and its clinical significance: a retrospective study. *OncoImmunology*.

[31] Li N., Li B., Zhan X. (2021). Comprehensive analysis of tumor microenvironment identified prognostic immune-related gene signature in ovarian cancer. *Frontiers in Genetics*.

